# Synergistic Activity of Colistin in Combination With Resveratrol Against Colistin-Resistant Gram-Negative Pathogens

**DOI:** 10.3389/fmicb.2018.01808

**Published:** 2018-08-07

**Authors:** Antonio Cannatelli, Silvia Principato, Olga L. Colavecchio, Lucia Pallecchi, Gian Maria Rossolini

**Affiliations:** ^1^Department of Medical Biotechnologies, University of Siena, Siena, Italy; ^2^SOD Genetic Diagnostic, Florence Careggi University Hospital, Florence, Italy; ^3^Department of Experimental and Clinical Medicine, University of Florence, Florence, Italy; ^4^Clinical Microbiology and Virology Unit, Florence Careggi University Hospital, Florence, Italy

**Keywords:** colistin, resveratrol, colistin resistance, antibiotic resistance breakers, combination therapy

## Abstract

**Objectives:** In this study, we investigated the antimicrobial activity of resveratrol in combination with colistin, a last-resort agent for the treatment of severe infections caused by multidrug resistant Gram-negative pathogens.

**Methods:** The synergistic activity and the bactericidal activity of colistin in combination with resveratrol was investigated by checkerboard assays and time-kill assays, respectively. A total of 21 strains were investigated, including 16 strains of different species (*Klebsiella pneumoniae, n* = 6, *Escherichia coli, n* = 6; *Citrobacter braakii, n* = 1; *Stenotrophomonas malthophilia, n* = 1; *Enterobacter cloaceae, n* = 1*; Acinetobacter baumannii, n* = 1) with acquired colistin resistance, three colistin-susceptible *K. pneumoniae* precursors, and two strains of intrinsically colistin-resistant species (*Serratia marcescens, n* = 1; *Proteus mirabilis, n* = 1). Mechanisms of acquired colistin resistance included chromosomal mutations (i.e., *mgrB, pmrAB*) and plasmid genes (*mcr-1, mcr-1*.2).

**Results:** Resveratrol did not show any significant intrinsic antimicrobial activity. Overall, a relevant synergistic antimicrobial activity of resveratrol in combination with colistin was observed with all tested strains, except for the three colistin-susceptible *K. pneumoniae* strains, and for two *mcr-1*-positive *E. coli* strains. In time-kill assays, performed with 15 selected strains, the combination of colistin 2 mg/L plus resveratrol 128 mg/L was bactericidal with 11 strains, and bacteriostatic for the remaining ones.

**Conclusions:** Resveratrol was found to potentiate colistin activity against a wide panel of colistin-resistant strains, regardless of species and resistance mechanisms, which would deserve further investigation for potential clinical applications.

## Introduction

Resveratrol (3,5,4′-trihydroxy-trans-stilbene) is a stilbenoid compound found in numerous plants. Resveratrol has been investigated for potential therapeutic effects in various diseases (Chen et al., 2005; Albani et al., 2010; Sawda et al., 2010; Sun et al., 2010; Singh et al., 2014; Li et al., 2016, 2017) and has also shown the potential for antiviral (Abba et al., 2015; Lin et al., 2017a,b) and antibacterial activity against some pathogens, including *Helicobacter pylori, Propionibacterium acnes*, and *Staphylococcus aureus* (Mahady et al., 2003; Su et al., 2014; Taylor et al., 2014). Anti-oxydant activity and interaction with various molecular targets, including kinases, sirtuins, and cytokines, have been suggested as mechanisms responsible for resveratrol activity, although knowledge on this aspect remains limited (Kuršvietiene et al., 2016).

Polymyxins are old antibiotics that, until recently, were rarely used in the clinical setting except for the practice of Selective Digestive Decontamination (SDD), carried out in some ICU settings to reduce infections caused by microorganisms from oropharyngeal and gastrointestinal tracts (Abis et al., 2013; Bar-Yoseph et al., 2016; Rawson et al., 2016). Recently, due to the emergence of extremely drug resistant (XDR) strains of Gram-negative pathogens, such as carbapenem-resistant *Enterobacteriaceae* (CRE) and carbapenem-resistant *Acinetobacter* sp. (CRA), polymyxins have regained a major role as last-resort agents for these infections, and their consumption has remarkably increased (Falagas and Kasiakou, 2005; Kaye et al., 2016). Unfortunately, also polymyxin resistance has emerged and is now increasingly reported, especially among CRE and CRA (Cannatelli et al., 2013; Monaco et al., 2014; Granata and Petrosillo, 2017; Jeannot et al., 2017; Nowak et al., 2017), further narrowing the treatment options.

In this study, we have tested the *in vitro* activity of resveratrol, alone and in combination with colistin, against a collection of colistin-resistant (COL-R) Gram-negative pathogens of different species. Despite the lack of any significant intrinsic antimicrobial activity, resveratrol exhibited a strong synergistic effect with colistin against many COL-R strains of different species, including *Escherichia coli, Klebsiella pneumoniae, Enterobacter cloacae, Stenotrophomonas maltophilia, Citrobacter braakii*, and also enterobacterial species that are naturally resistant to polymyxins (e.g., *Proteus mirabilis* and *Serratia marcescens*).

## Materials and methods

### Bacterial strains

Bacterial strains investigated in this work are listed in Table 1. These included 18 COL-R strains of different species (*A. baumannii, K. pneumoniae, E. coli, E. cloacae, S. maltophilia, C. braakii, P. mirabilis*, and *S. marcescens*) and three colistin-susceptible (COL-S) *K. pneumoniae* that were precursors of three COL-R strains. For *S. maltophilia*, for which clinical breakpoints for colistin are not available, the definition as COL-R was arbitrarily based on the high-level colistin MIC (i.e., 32 mg/L) as compared with the colistin MIC distribution for the species (Sergio et al., 2017). For some strains, the mechanism of colistin resistance had been previously characterized (Table 1).

**Table 1:** Results of checkerboard assays of colistin in combination with resveratrol.

**Strains**	**Source**	**Phenotype**	**ST**	**Reference**	**Mechanism of colistin resistance**	**Colistin MICs (mg/L) at different resveratrol concentrations (mg/L)**						
						**Resveratrol concentration (mg/L)**						
						**0**	**8**	**16**	**32**	**64**	**128**	**256**
*E. coli* LC711/14	Urine	COL-R	ST59	Cannatelli et al., 2017	PmrB Leu_10_Pro	8	4	2^*^	1^*^	0.25^*^	0.25^*^	0.125^*^
*E. coli* LC761/12	Urine	COL-R	ST131	This study	PmrA Asp_82_Asn^c^	4	0.5^*^	0.5^*^	0.25^*^	0.125^*^	0.125^*^	0.125^*^
*E. coli* FI-4451	Urine	COL-R	ST117	Cannatelli et al., 2016	*mcr-1*	8	8	8	4	4	4	4
*E. coli* FI-4531	Urine	COL-R	ST648	Cannatelli et al., 2016	*mcr-1*	8	4	4	4	4	2^*^	2^*^
*E. coli* FI-4592	Urine	COL-R	ST804	Cannatelli et al., 2016	*mcr-1*	8	4	4	4	4	4	4
*E. coli* LC902/14	Urine	COL-R	ST602	Cannatelli et al., 2016	*mcr-1*	8	4	4	4	4	2^*^	2^*^
*C. braakii* CA-26	Food	COL-R	–	Sennati et al., 2017	*mcr-1*	8	4	4	4	4	2^*^	2^*^
*S. maltophilia* 157	–	COL-R	n.d.	This study	n.d.^d^	32	4	2^*^	1^*^	0.5^*^	0.125^*^	0.125^*^
*E. cloacae* CIP6085	–	COL-R	n.d.	–	n.d.^e^	128	128	32^*^	8^*^	0.5^*^	0.25^*^	0.125^*^
*K. pneumoniae* KKBO-1^a^	Blood	MDR/COL-S	ST258	Cannatelli et al., 2013	–	0.5	0.5	0.5	0.5	0.5	0.5	0.5
*K. pneumoniae* KKBO-4	Blood	MDR/COL-R	ST258	Cannatelli et al., 2013	IS*5-like* at nt.75 of *mgrB*	64	64	64	16^*^	8^*^	4^*^	4^*^
*K. pneumoniae* KPB-1^a^	Blood	MDR/COL-S	ST512	Cannatelli et al., 2014a	–	0.5	0.5	0.5	0.5	0.5	0.5	0.5
*K. pneumoniae* KPB-2	Blood	MDR/COL-R	ST512	Cannatelli et al., 2014a	PmrB Leu_82_Arg	4	4	4	4	2	1^*^	0.5^*^
*K. pneumoniae* KK207-1^a^	Blood	MDR/COL-S	ST258	This study	–	0.5	0.5	0.5	1	0.5	0.5	0.5
*K. pneumoniae* KK207-2	Blood	MDR/COL-R	ST258	Cannatelli et al., 2014b	IS*5-like* at nt.75 of *mgrB*	64	64	64	64	4^*^	1^*^	0.5^*^
*K. pneumoniae* 6884	Blood	MDR/COL-R	ST512	Di Pilato et al., 2016	*mcr-1.2*	8	8	8	8	4	1^*^	1^*^
*K. pneumoniae* KPFan^b^	–	COL-R	ST674	Cannatelli et al., 2015	IS*102-like* at nt.69 of *mgrB*	32	32	16	8^*^	2^*^	1^*^	1^*^
*K. pneumoniae* KPGP1^b^	–	COL-R	ST16	Cannatelli et al., 2015	IS*kpn14-like* at nt.124 of *mgrB*	32	32	32	32	2^*^	1^*^	1^*^
*A. baumannii* N50	Respiratory tract	MDR/COL-R	ST2	D'Andrea et al., 2009	IS*Ava1* at nt. 531 of *pmrB*	64	64	64	64	8^*^	1^*^	1^*^
*S. marcescens* CCUG1647^T^	–	COL-R	n.d.	–	Naturally resistant	>128	>128	>128	>128	16^*^	1^*^	1^*^
*P. mirabilis* NO-051	Cutaneous ulcer	COL-R	n.d.	D'Andrea et al., 2006	Naturally resistant	>128	>128	>128	>128	>128	>128	8^*^

a These strains were the COL-S precursors of COL-R K. pneumoniae KKBO-4, K. pneumoniae KPB-2, and K. pneumoniae KK207-2 strains, respectively. Resveratrol MICs were >512 mg/L for all tested strains.

b These COL-R strains were selected in vitro, using two COL-S precursors (Cannatelli et al., 2015). Multidrug-resistant phenotypes (MDR) refer to strains resistant to carbapenems (imipenem and meropenem), ciprofloxacin, and amikacin. n.d. = not determined.

c Colistin resistance in E. coli LC761/12 was putatively associate to PmrA Asp_82_Asn novel allelic variant, being absent all other known mechanisms of acquired colistin resistance in E. coli (data not shown).

d The colistin resistance mechanism in this strain is unknown.

e Enterobacter CIP6085 was found to be negative for mcr-1 and mcr-2 detection. The colistin resistance mechanism in this strain is unknown.

* *Combinations in which colistin/resveratrol combinations yielded a synergistic activity (FICI ≤ 0.5). The lower concentration of resveratrol needed for restoring susceptibility to colistin is shaded in gray*.

### Chemicals

Colistin sulfate and resveratrol were obtained from Sigma-Aldrich (Saint Quentin Fallavier, France). Resveratrol (Thermo Fisher, Germany) was dissolved in dimethyl sulfoxide (DMSO) (Sigma-Aldrich, Saint Louis, USA) at a concentration of 20 mg/mL.

### *In vitro* susceptibility testing, checkerboard assays, and time-kill assays

MICs of colistin and resveratrol were determined by reference broth microdilution (Clinical and Laboratory Standards Institute, 2015) using cation-adjusted Mueller-Hinton broth (MHB) (bioMérieux, Florence, Italy). Colistin MICs were interpreted accordingly to the EUCAST clinical breakpoints, version 8.0 (www.eucast.org). Checkerboard assays to test the antimicrobial activity of combinations of colistin plus resveratrol were carried out as described previously (Tascini et al., 2013), using MHB and 96-well microtiter plates (Sarsted, Nümbrecht, Germany). Each well was inoculated with 50 μl of a suspension of 5 × 10^5^ CFU/mL of the test strain in a final volume of 100 μl. Inocula were prepared by direct suspension in MHB of bacteria grown overnight onto MH agar plates. Results were read after incubation at 35°C for 16–20 h and interpreted as follows: FICI ≤ 0.5, synergism; FICI > 4.0 antagonism; FICI 0.5–4 no interaction. Data were obtained in at least two independent experiments.

Time–kill assays were performed in duplicate, by inoculating 5 × 10^6^ CFU of each strain into 2 mL of MHB in 24 Deep Well RB Block (Thermo Fisher Scientific, MA USA), at 35°C, under static condition (Clinical and Laboratory Standards Institute, 2015). CFU counts were determined at different time points, by plating appropriate dilutions onto LB Agar (Sezonov et al., 2007).

In time kill assays, the DMSO concentration remained always below 1% (v/v), as recommended by CLSI guidelines (Clinical and Laboratory Standards Institute, 2015). In MIC testing and checkerboard assays, the conditions with resveratrol concentrations of 256 and 512 mg/L contained DMSO concentrations higher than 1% (i.e., 1.36 and 2.72%, respectively). Appropriate controls to exclude any potential synergistic activity between colistin and DMSO were always included.

## Results and discussion

### Synergistic activity of colistin in combination with resveratrol in checkerboard assays

A collection of 21 strains of eight different Gram-negative species were tested for susceptibility to resveratrol, colistin, and combinations thereof. The collection included 15 COL-R strains of species that are naturally susceptible to colistin (*C. braakii, E. coli, K. pneumoniae, E. cloacae, A. baumannii*), two COL-R strains of naturally resistant species (*S. marcescens* and *P. mirabilis*), and one *S. maltophilia* strain with high colistin MIC (that was considered COL-R for the purpose of this work). It also included three COL-S strains of *K. pneumoniae*, which were the precursors of three of the COL-R strains (Table 1).

MICs of resveratrol were >512 mg/L for all tested strains, showing the lack of any intrinsic antimicrobial activity of resveratrol alone against these Gram-negative pathogens.

Checkerboard assays revealed a clear dose-dependent synergistic activity of resveratrol with colistin vs. COL-R strains of different species, including intrinsically resistant species such as *S. marcescens* and *P. mirabilis*. Synergism was not observed with two of the four COL-R *E. coli* strains carrying the *mcr-1* determinant and with the COL-S *K. pneumoniae* precursors of three COL-R strains (Table 1).

When synergism was evident, resveratrol was able to decrease colistin MICs to values equal or lower than the susceptibility breakpoint (i.e., 2 mg/L) in most cases, at concentrations variable from 8 to 128 mg/L. In particular, this was the case with four of the six COL-R *E. coli*, with five of the six COL-R *K. pneumoniae*, with the COL-R *C. braakii*, with the COL-R strains of *A. baumanni, E. cloacae* and *S. maltophilia*, and with the type strain of *S. marcescens*. The synergistic effect was observed in presence of different colistin resistance mechanisms and with strains of different clonal lineages, including representatives of known high risk clones (e.g., ST131 and ST59 for *E. coli*, or ST512 and ST258 for *K. pneumoniae*; Table 1).

### Synergistic activity of resveratrol and colistin in time-kill assays

In order to investigate if colistin in combination with resveratrol had a bactericidal effect, time-kill assays were carried out with the 15 COL-R strains for which checkerboard assays had showed a synergistic effect. The colistin concentration used in time-kill experiments corresponded to the clinical breakpoint for susceptibility (2 mg/L), or to 0.5 × MIC and 1 × MIC, while the resveratrol concentration used was 128 mg/L, which was able to inhibit the growth in most cases when combined with colistin at 2 mg/L (Table 1).

The time-kill assays showed a bactericidal activity (i.e., a reduction ≥3 log_10_ of the initial bacterial inoculum) of resveratrol 128 mg/L in combination with colistin 2 mg/L with 11 of the 15 COL-R strains tested, while with four strains (*E. coli* FI-4531, *K. pneumoniae* KKBO-4, *K. pneumoniae* KK207-2, *A. baumannii* N50) the combination exerted a static effect (Figure 1). Overall, with these strains when colistin was used at 0.5 X MIC and 1 X MIC in combination with resveratrol 128 mg/L, a bactericidal effect was observed, except for *E. coli* FI-4531, in which this combinations seem to be less effectives (Figure 2).

**Figure 1:** Time-kill assays with colistin 2 mg/L in combination with resveratrol 128 mg/L. Data are mean values from the results of two independent experiments, and the error bars represent standard deviations. The lowest number of CFU (detection limit) that can be detected by the method used is 1E+02 CFU/mL.

**Figure 2:** Time-kill assays with colistin at 0.5 or 1 X MIC in combination with resveratrol 128 mg/L, in the strains in which colistin 2 mg/L plus resveratrol 128 mg/L yielded a bacteriostatic effect. Data are mean values from the results of two independent experiments, and the error bars represent standard deviations. The lowest number of CFU (detection limit) that can be detected by the method used is 1E+02 CFU/mL.

Altogether, the results were consistent with data obtained in checkerboard assays (Table 1). In fact, all strains exhibiting a colistin MIC <1 mg/L or >2 mg/L in combination with resveratrol 128 mg/L, showed a bactericidal or bacteriostatic effect in time-kill curves, respectively. On the other hand, a variable effect was observed with strains for which, in the presence of resveratrol 128 mg/L, colistin MIC was lowered to 2 or 1 mg/L (Figure 1).

Considering the diversity of species tested, (*C. braakii, E. coli, K. pneumoniae, E. cloacae, S. marcescens, A. baumannii, S. maltophilia*) expressing different colistin resistance mechanisms, the “cidal/static” activity of colistin 2 mg/L in combination with resveratrol 128 mg/L did not appear to be dependent on species or the resistance mechanism.

The absence of any synergistic activity with COL-S strains could suggest a likely resveratrol interaction with the lipid A modification systems that are responsible for colistin resistance in COL-R strains. However, the mechanism of synergism observed between resveratrol and colistin with COL-R strains remains unknown and will be the subjects of further investigations.

## Concluding remarks

MDR and XDR Gram-negative bacteria (e.g., CRE and CRA) have been increasingly reported worldwide (Cannatelli et al., 2013; Monaco et al., 2014), and are listed among resistant pathogens with the highest priority for research and development of new antibiotics by the WHO (WHO, 2017).

Colistin remains one of the few antibiotics active against these pathogens, and represents a drug of last resort for the treatment of CRE and CRA severe infections (Falagas and Kasiakou, 2005; Kaye et al., 2016). It is also used for the Selective Digestive Decontamination (SDD) in combination with other agents (i.e., tobramycin, amphotericin B) (Abis et al., 2013; Rawson et al., 2016), and is increasingly administered for the management of chronic lung colonization by *Pseudomonas aeruginosa* in cystic fibrosis (Sherrard et al., 2014). In this perspective, the increasingly dissemination of colistin resistance in these pathogens represents a matter of public health concern (Cannatelli et al., 2013; Monaco et al., 2014; Granata and Petrosillo, 2017; Jeannot et al., 2017; Nowak et al., 2017).

This worrisome scenario has forced the scientific community to evaluate new therapeutic approaches to face the antibiotic resistance crisis. One promising strategy is offered by non-antibiotic drugs which overcome the resistance mechanism (Antibiotic Resistance Breakers; ARB) when combined with failing antibiotics (Brown, 2015). A well-proven example of such approach is represented by the new beta-lactamase inhibitors (i.e., avibactam, vaborbactam; Giani et al., 2016). Nonetheless, considering the multitude of resistance determinants and their rapid evolution potential, additional solutions must be implemented. Among the diverse approaches investigated over the last years, some natural compounds (i.e., resveratrol, quercetin, curcumin, pterostilbene), which have shown anti-bacterial properties (Su et al., 2014; Taylor et al., 2014; Hwang and Lim, 2015; Kuršvietiene et al., 2016; Zhou et al., 2018), could also be of interest.

In this work we provided the first *in vitro* demonstration that resveratrol can act as an ARB, potentiating colistin activity against a collection of COL-R Gram-negative pathogens, covering a wide panel of species and colistin resistance mechanisms. A limitation of this study was that the synergism between resveratrol and colistin was not tested with COL-R strains of *P. aeruginosa*, which at the time of the study were not available in our collection.

The potential to exploit this feature *in vivo* could depend on the resveratrol concentrations achievable *in vivo*, at different body sites. A number of pre-clinical and clinical studies have previously investigated resveratrol administered orally (Tomé-Carneiro et al., 2013), intravenously (Tomé-Carneiro et al., 2013), or by inhalation (Varricchio et al., 2014), but current knowledge on resveratrol pharmacokinetics in humans remain limited. When given orally, resveratrol is absorbed but readily metabolized, leading to a rather low bioavailability (Walle et al., 2004; Boocock et al., 2007; Tomé-Carneiro et al., 2013), while the non-absorbed fraction can be transformed by components of the gut microbiota (Tomé-Carneiro et al., 2013). Several resveratrol-derived metabolites have been identified in human and animals following oral or parenteral administration, including trans- and/or cis- forms of mono- and diglucuronides, mono- and disulfates, sulfoglucuronides, and dihydroresveratrol metabolities, which undergo renal and fecal excretion (Walle et al., 2004; Boocock et al., 2007; Tomé-Carneiro et al., 2013).

Consider that the activity of specific circulating resveratrol metabolites is still under debate, and the concentration of unchanged resveratrol in human urine, feaces and plasma has still not been clearly determined, the use of colistin/resveratrol combinations for Selective Digestive Decontamination or treatment of urinary and systemic infections would deserve further investigation.

The most promising setting to exploit the synergism between resveratrol and colistin would be that of respiratory tract infections, where the administration of inhaled formulations of resveratrol might overcome the issues related to low bioavailability and metabolism of this compound. Being resveratrol also administered by nebulization in humans (Varricchio et al., 2014), the potential efficacy of colistin/resveratrol inhaled formulations could deserve further attention, especially in cases of chronic lung colonization by difficult-to-treat Gram-negatives, such as in cystic fibrosis, chronic obstructive pulmonary disease or bronchiectasis not related to cystic fibrosis.

Present results represent a proof of principle for further studies aimed at evaluating the potential role of resveratrol as colistin ARB in other *in vitro* (e.g., biofilm susceptibility testing) and *in vivo* models (e.g., Selective decontamination of the digestive tract).

- “The content is object of Italian Patent Application No. 102017000025738 filed on 08.03.2017”
- “The content is object of International Patent Application No. PCT/EP2018/055595 filed on 22.05.2018.”

## Author contributions

AC, LP and GR: study design, data analysis or interpretation, manuscript preparation. AC, SP, and OC: experimental studies, statistical analysis.

### Conflict of interest statement

The authors declare that the research was conducted in the absence of any commercial or financial relationships that could be construed as a potential conflict of interest. The reviewer MB and handling Editor declared their shared affiliation.
